# Effectiveness and Safety of High-Power Radiofrequency Ablation Guided by Ablation Index for the Treatment of Atrial Fibrillation

**DOI:** 10.1155/2022/5609764

**Published:** 2022-08-12

**Authors:** Xuefeng Zhu, Chunxiao Wang, Hongxia Chu, Wenjing Li, Huihui Zhou, Lin Zhong, Jianping Li

**Affiliations:** ^1^Department of Cardiology, The Affiliated Yantai Yuhuangding Hospital of Qingdao University, China; ^2^Department of Ultrasound Medicine, The Affiliated Yantai Yuhuangding Hospital of Qingdao University, China; ^3^Department of Pathology, The Affiliated Yantai Yuhuangding Hospital of Qingdao University, China

## Abstract

**Background:**

To investigate the efficacy and safety of ablation index- (AI-) guided high-power radiofrequency ablation in the treatment of atrial fibrillation (AF).

**Methods:**

Outcomes of radiofrequency (RF) applications were compared in a swine ventricular endocardial model (*n* = 10 each for 50 W, 40 W, and 30 W; AI = 500). And a total of 100 consecutive patients with paroxysmal AF undergoing pulmonary vein isolation (PVI) were included. The patients were divided into two groups (*n* = 50 for each) as follows: control group, treated with conventional power (30 W) ablation mode; and study group, treated with high power (40 W) radiofrequency ablation mode. All groups were treated with the same AI value guided the ablation (target AI = 400/500 on posterior/anterior wall, respectively). Acute pulmonary vein (PV) reconnection was assessed post adenosine administration 20 minutes after ablation. Subsequently, pathological observation of porcine heart lesions and necrotic tissue was performed. Additionally, statistical analyses were carried out on patients' baseline clinical characteristics, surgical data, and total RF energy.

**Results:**

In swine ventricular endocardial RF applications, compared with 40 W and 30 W, the use of 50 W was associated with shallower tissue lesion depth (*p* < 0.001) and greater lesion maximum diameter (*p* < 0.001). Compared with 40 W and 30 W, tissue necrosis caused by 50 W was the deepest and largest (*p* < 0.001). In pulmonary vein isolation (PVI), there was no significant difference in baseline data between the study group and control group (*p* > 0.05). In patients with paroxysmal atrial fibrillation, the procedure time in the high-power group was significantly shortened (*p* < 0.001). The ablation time was significantly shorter (*p* < 0.001). Compared with control group, RF energy per point and acute pulmonary vein (PV) reconnection were lower (*p* < 0.001), and first-pass PVI was higher (*p* < 0.01) in study group. There were no significant differences in complications and sinus rhythm maintenance at 12 months between the two groups (*p* > 0.05).

**Conclusions:**

Compared with conventional (30 W) PVI, AI-guided high-power (40 W) was safe and associated with shorter procedure time and reduced acute PV reconnection.

## 1. Introduction

Radiofrequency (RF) ablation is widely used in the treatment of patients with atrial fibrillation (AF) via transmural, continuous, and lasting lesion formation with pulmonary vein isolation (PVI). Despite optimization of RF current transfer, RF energy transfer duration, catheter contact forces (CF), and catheter stability [1], pulmonary vein (PV) reconnection occurs acutely and at 3 months after PVI at a frequency of 22% and 15%, respectively [2, 3], mainly secondary to reversible damage, partial thickness, and/or incomplete ablation [4–6]. In recent years, the ablation index (AI) has been widely applied to treat drug-resistant paroxysmal AF [7]. AI is known as a novel quantitative ablation lesion marker that combines contact force (CF), time, and power in a weighted formula [8, 9]. In recent studies, patients undergoing AI-guided ablation of AF have good clinical outcomes, and the procedure time and ablation time are relatively short; meanwhile, it is considered a feasible and safe technique [7, 10, 11].

Traditional RF ablation typically employs low power long duration (LPLD) ablation (25-35 W), which is intended to produce mature ablated lesions and minimize complications [12, 13]. However, high-power ablation consistently resulted in shorter procedural times, reduced fluoroscopy dose, and decreased total RF energy delivery [14, 15]. Furthermore, high-power short-duration (HPSD) RF ablation is resistive heating and is more suitable for wide, continuous lesions while reducing complications associated with posterior wall isolation (PWI) [13, 16]. For example, Bhaskaran et al. [17] indicated that HPSD (50 W/5 seconds and 60 W/5 seconds) is as safe and effective as LPLD (40 W/30 s), with increased transmission and fewer complications. Winkle et al. [18] indicated that shorter duration 50 W lesions has been associated with better long-term outcomes without an increase in rates of complications. Additionally, high-power (40-50 W) RF ablation under the guidance of unipolar signal modification displays higher first-pass PVI and guarantees a robust one-year efficacy [19]. In recent animal studies, 50 W/5 seconds was superior to LPLD ablation for lesion creation with lower complication rates [17, 20]. In AI-guided high-power (50 W) ablation, the time to complete PVI is shorter, with higher first-pass isolation rate, lower left atrial- (LA-) PV reconnection rate, and no increase in complications, so it is considered a safe and feasible ablation technique [9, 21–23]. But reports on the safety and efficacy of AI-guided high-power RF ablation for paroxysmal atrial fibrillation are warranted.

In the present 2-tiered study, we first tested in a swine model the effect of different power outputs on lesion creation at the ventricular level and compared lesion dimensions for the same AI value. A clinical study then assessed whether AI-guided high-power ablation relative to AI-guided standard power ablation is relevant for PVI in cases of paroxysmal atrial fibrillation.

## 2. Methods

The present study was divided into 2 successive parts. An animal study provided efficacy and safety data, which oriented the clinical study for the choice of RF duration. The 2 parts followed the same technical principles for clinical research.

### 2.1. Animal Study

Swine hearts were obtained from an approved vendor (Shandong Animal Experiment Center) and studied at a laboratory of Yantai Yuhuangding Hospital. After pericardium excision, hearts were placed in a tissue bath with circulating arterial blood at a rate of 200 ml/min and temperature of 37°C within the thigh preparation chamber. Arterial blood was extracted (400 ml), and unfractionated heparin was added to maintain an activated clotting time of 350 to 400 s. Individual RF applications were performed at the endocardial aspect of the ventricles. RF ablation was performed with a 3.5 mm-tip open-irrigated contact force-sensing catheter (ThermoCool Smart Touch (ST), Biosense Webster, South Diamond Bar, USA). The catheter was positioned perpendicular to the left ventricular tissue and adjusted by the operator maintaining a constantly desired contact-force (CF) of 10 g throughout energy delivery. For the same AI of 500, power output was 30 W for the control lesions and 40 W and 50 W for the study lesions, respectively, at ten ablation points. Ablation sites were > 10 mm apart to avoid any lesion overlap and to facilitate histopathologic evaluation. Lesions and necrotic areas were then bisected in two perpendicular planes to measure depth and maximal internal width. After proper fixation in 10% natural buffered formalin, hearts were trimmed to isolate all ablation sites, which were processed and embedded in paraffin. All paraffin blocks were subjected to microtome dissection twice serially at 5 *μ*m, before being stained with hematoxylin and eosin for histopathologic analysis.

### 2.2. Clinical Study

#### 2.2.1. Patient Population

The subjects were consecutive symptomatic patients with paroxysmal AF undergoing initial point-by-point RF ablation at Yantai Yuhuangding Hospital (Yantai, China) from April 2018 to February 2019. A total of 100 patients were included and randomly divided into the study group (*n* = 50) and the control group (*n* = 50). The control group was treated with standard power (30 W), whereas the study group was treated with high-power (40 W). Study exclusion criteria were left atrial thrombus, age < 18 years, prior AF ablation, left ventricular ejection fraction < 35%, severe valvular or coronary artery disease, thyrotoxicosis, and left atrial diameter > 60 mm. All patients provided written informed consent for the ablation procedure. The Ethics Committee of Yantai Yuhuangding Hospital (Yantai, China) approved the protocol of the present study.

### 2.3. Ablation Protocol

Our periprocedural anticoagulation protocols have been previously described [24]. The procedure was performed under local anesthesia consisting of lidocaine administration in the groin and left subclavian region and fentanyl as an analgesic. The CARTO3 system (Biosense Webster, Diamond Bar, USA) was used in all cases for 3D mapping. First, one 6F decapolar catheter was positioned in the coronary sinus, followed by double transseptal punctures, 2 SL1 (8 F, Abbott, USA) sheaths were inserted into the LA, one for the multipolar mapping catheter to map the anatomy of the LA and the other for the 3.5 mm tip open-irrigated contact force-sensing catheter. After creating an anatomical CARTO map of the left atrium, the borders of all four pulmonary veins (PVs) were marked on the CARTO map. The patient underwent systemic anticoagulation with intravenous heparin during surgery to maintain an activated clotting time > 300 seconds.

Next, all 4 PVs underwent encirclement by point-by-point RF applications (target AI was 400 for the posterior segment, and 500 elsewhere) and other ablations as clinically indicated (Figure 1). RF applications were performed with power-control mode, temperature limited to 45°C, and saline irrigation (17 to 30 mL/min). Ablation was delivered aiming for a CF of 10-20 g. The procedural endpoint was PVI. The entrance block was confirmed by the absence of PV potentials recorded with the tissue proximity instruction (TPI) of pentaray catheter [25]. Exit block was defined as the failure to capture the left atrium while pacing with the TPI of pentaray catheter within the antrum carina included [26]. In both groups, a total of 20 minutes waiting period was observed following PVI, after which 18 mg of adenosine was administered for each PV with the pentaray positioned to record any PV reconnection. The AI Software Module (Biosense Webster, Diamond Bar, CA) was used for determination of Automatic lesion tagging (VISITAG). Ablation was delivered with ST catheters in power-controlled mode with 40 W in study group and 30 W in the control group. The “distance ruler” function was used on CARTO; it shows a continuous measure of the distance from the center of the last VISITAG which changes in real-time (Figure 1). This distance was kept <6 mm when commencing an ablation lesion. VISITAGs were displayed showing ablation lesions with 3 mm radius so that VISITAGs < 6 mm apart could be seen to overlap (Figure 1). After the circumferential line of ablation was completed, the geometry was made transparent to look for any gaps between VISITAGs (which would indicate a gap > 6 mm). If any gaps were seen, they were filled with an ablation lesion. If any VISITAGs were not red (indicating that they had not met their regional AI target), then, it was left at the operator's discretion as to whether to repeat the lesion. Only after the circumferential line of ablation was completed, if the PV was not isolated, further ablation was guided by the pentaray catheter delivered either on the circumferential line of ablation where there was signal or just within it. Ablation was not delivered within the PVs or on the intervenous ridge between PVs unless PV isolation could not be achieved without doing so. First-pass antral isolation designated exit block obtained after initial anatomic encirclement. The information on drugs and equipment used in this study are shown in Table 1.

### 2.4. Data Collection and Analysis

For each patient, we recorded age, gender, CHADS_2_ ((congestive heart failure, hypertension, age ≥ 75 years), and diabetes, previous stroke (double weight)) and CHA_2_DS_2_-VASc (congestive heart failure, hypertension, age ≥ 75 years (double weight), diabetes, previous stroke (double weight), vascular disease, age 65–74 years, and female sex category) scores, body mass index (BMI), LA size, prior strokes/transient ischemic attacks (TIAs), and the presence of hypertension, diabetes, coronary artery disease (CAD), cardiomyopathy, and obstructive sleep apnea. For each ablation, we determined procedural, total RF times, and CF. Complications were reported on a per-procedure basis. Complications examined were death, incidence of pericardial tamponade, strokes occurring within 48 hours, strokes occurring from 48 hours–30 days, and PV stenosis requiring intervention, phrenic nerve paralysis, atrioesophageal fistulas, steam pops, and catheter char. Procedure time was defined as time from the first ablation point to PVI, not including additional ablation beyond PVI. The RF time was defined as the time for which RF energy was applied. Primary outcome measures were defined as no AF, atrial flutter, or atrial tachycardia (AT) lasting more than 30 seconds off antiarrhythmic drugs after a 3-month blanking period.

### 2.5. Follow-Up

All patients were discharged home within 48 to 72 hours. Vitamin K antagonists or direct oral anticoagulants were prescribed for at least 2 months (subsequent strategy depending on the CHA2DS2-VASc score). Patients were followed up in clinic with an ECG at 3 and 9 months with 24 hours. Holter monitoring was performed at 6 and 12 months and beyond as dictated by symptoms.

### 2.6. Statistical Analysis

For each part of the study, variables are presented as mean ± SD or percentages, as appropriate. Continuous and categorical data were compared with the Student *t* test (two-tailed) and the *χ*^2^ test (or Fisher exact test in case of small sample), respectively. *p* < 0.05 was considered as statistically significant.

## 3. Results

### 3.1. Animal Study

Table 2 shows a comparison of lesions and necrosis in control (30 W) and study (40 W, 50 W) swine hearts for a total of 30 RF applications. By visual inspection, 50 W use was associated with shallower lesions; and increasing RF power and shortening RF duration yielded greater maximum diameter (green line) and larger and deeper tissue necrosis area (red line) and nuclear pyknosis by histopathology (Figure 2).

### 3.2. Clinical Study

Since there was a small amount of scab on the catheter tip during ablation at 50 W in animal experiments, we chose 40 W as the high-power ablation in the clinical study. A total of 100 consecutive patients with paroxysmal AF were evenly distributed to control group (first 50 patients) and study group (last 50 patients); their baseline clinical characteristics are summarized in Table 3. A total of 8726 RF lesions were delivered in these 100 patients, and procedural data are summarized in Table 4.  Figure 3 shows the distribution of lesions by ranges of CF. The study vs. control group had shorter total procedure time (*p* < 0.001), left and right encirclement procedure time (*p* < 0.001), total ablation time required for PVI (*p* < 0.001), ablation time per point in different parts of PV, and total RF energy delivered per procedure (*p* < 0.001; Figure 4).  Figure 5 shows the energy delivery per point throughout PV. First-pass isolation was more frequent in the study group (*p* < 0.01), occurring in both left and right in 70% PVs (35/50) of study patients vs. 42% (21/50) of controls (*p* < 0.001). The study vs. control group required fewer additional ablations on the intervenous ridge between the PVs to isolate them (*p* < 0.001), and had fewer acute PV reconnections (*p* < 0.001).

At mean 1.04 ± 0.62 years follow-up, the percentage of patients free from AF/AT after a single procedure was 92% (46/50) in the study group and 84% (42/50) in the control group (*p* = 0.22). There were no cases of stroke, TIA, pericardial tamponade, atrial-esophageal fistulae, PV stenosis, or death.

## 4. Discussion

In the present study, two-tiered animal and clinical study yielded four major findings. First, in swine hearts, higher vs. lower power RF applications were more effective in creating larger and deeper necrosis yet shallower lesions, while lower power was associated with deeper lesions without basophilic changes in connective tissue. Second, in patients with paroxysmal AF, high-power ablation was associated with shorter procedure times and less total RF energy delivery, especially on the left anterior wall. Third, AI, the novel marker incorporating contact force-time power, reliably predicted the degree of necrosis in RF delivery. Fourth, higher power combined with AI increased PVI effectiveness with more frequent first-pass isolation, decreased acute reconnection, and favorable 12-month outcomes.

### 4.1. High-Power Ablation

Myocardial lesion creation starts at 45°C, being partially reversible below 50°C (transient stunning), and definitive above 50°C (durable necrosis) [27]. RF energy delivery to tissue is a complex interaction [1]. Thermal injury induced by electrical current delivery with an irrigated-tip comprises resistive and conductive phases. Resistive heating, which probably occurs relatively early in the RF application, depends upon current delivered to the tissue and the resistance seen by the RF generator. Greater resistive heating can be achieved by the use of higher RF power or lower resistance. For instance, with standard power (25–30 W), temperature already rises above 50°C, but tissue necrosis is confined to the first 1 to 1.5 mm from the ablation catheter tip [28]. Conductive heating is secondary passive heating of deeper tissue which increases with longer duration RF applications. Tissue needs to be heated to 50°C or higher for several seconds to achieve irreversible coagulation necrosis which results in an electrically silent scar. Force sensing and stability monitoring have considerably facilitated the reproducibility of heat transmission to the tissue [29, 30]. Thus, the balance between power and duration parameters involved in resistive and conductive heating, respectively, has an increasing impact on lesion creation. By increasing resistive heating size, high-power (40–50 W) may theoretically be beneficial for the generation of durable lesions (temperature above 50°C) whose dimensions may be particularly suitable for PVI as antral thickness is consistently below 4 mm [31].

### 4.2. Animal Experiments

Conventional LPLD (25-35 W) ablation is used to generate mature ablated lesions and reduce complications [12, 13]. But recent studies have shown that HPSD is as safe and effective as LPLD while shortening the operative time, and it has a higher first-pass PVI rate and lower acute pulmonary vein reconnection (PVR) [17, 32, 33]. Additionally, Borne et al. [34] found using a porcine *in vivo* model that although a 50 W/5-second ablation is similar in volume to a 20 W/30-second ablation, it is shallower in depth while potentially causing less collateral damage. Hence, in this study, we divided the porcine left ventricle into control (30 W) and study groups (40 W and 50 W) and performed 30 RF applications followed by histopathological evaluation. Results indicated that 50 W power ablations for short durations at 10 g of CF created larger and deeper necrosis than that observed with 40 W and 30 W of power; however, the use of 30 W resulted in deeper lesions but without basophilic changes which might render them more susceptible to tissue recovery. HPSD applications were more effective in creating larger and deeper necrosis yet shallower lesions may be due to reduced temperature rise in deeper tissue relative to standard lesions. However, the area of tissue necrosis near the surface of the ablation catheter tip is larger because it is more dependent on resistive heating, which is proportional to power. The larger diameter of necrosis in study group might contribute to complete encirclement of pulmonary veins, by ensuring better contiguity with adjacent necrosis. At the same time, it was found that higher power (50 W) ablation may lead to more complete cell necrosis. However, nuclear pyknosis was observed only more superficially with low-power ablation, and only cell edema was present in the deep part, which may lead to cell reactivation and consequent acute and late PV reconnection and AF recurrence. Since there was a small amount of scab on the catheter tip during 50 W ablation in animal experiments, we chose 40 W as high-power ablation and 30 W as control ablation in the clinical study.

### 4.3. Clinical Research

#### 4.3.1. Procedural Time

In the present study, high-power ablation was associated with shorter procedural duration due to the shorter time required for lesion creation, more first-pass PVI, and fewer acute pulmonary vein reconnections. It is known that the first 10 seconds of RF application are the most important for lesion formation with diminishing effect beyond 20 seconds, and the ideal contact force is 10-20 g [32]. Nilsson et al. [15] reported that ablation with 45 W for 20 seconds vs. 30 W for 120 seconds was associated with shorter PV isolation time, mean fluoroscopy time, radiation dose, and total RF application time. In ventricles from freshly killed pigs, Goyal et al. [20] showed that for 20 g of CF, the time needed to create a 4 mm deep lesion decreased from just over 20 seconds for 20 W to 6–7 seconds for 50 W. In the present study, under the same pressure, the ablation time per point of the left atrial posterior wall in the high-power group was 8-9 seconds shorter than that in the control group and 10-13 seconds shorter for the left atrial anterior wall. Because catheter instability in a constantly beating heart may also account for the difficulty to transmit heat to the tissue, RF application time shortening probably optimizes lesion creation by increasing the likelihood of catheter stability throughout the entire RF application, particularly for ablation of the left atrial anterior wall by the left atrial appendage ridge. The significantly smaller pressure of <10 g (60%) used for the left atrial anterior wall than for the other three surfaces helps avoid catheter slippage (Figure 6). However, low power use requires longer time which increases catheter slippage, and the additional time spent adjusting the catheter may cause discontinuous ablation tissue edema, lower first-pass PVI rate, and increased risk of acute PV reconnections. In the present study, ablation time of the left anterior wall was longer than that of other parts of the left atrium in both study and control groups (Figure 7); however, it was shorter in the study than the control group likely secondary to shorter time required to adjust the catheter or the ineffective point of ablation (procedure time minus total ablation time).

### 4.4. AI Value

AI is a novel marker incorporating contact force, time, and power in a weighted formula. The use of contact force targets and markers of ablation output such as FTI reduces recurrence and complication rates in cohorts of patients with AF undergoing PVI [3, 35, 36]. Single-center studies on AI-guided ablation reported very high rates of first-pass PVI (97-98%) and very low rates of acute PV reconnection (2-6%) [36, 37]. In the present study on AI-guided high-power ablation, rates of first-pass PVI were high at 87% albeit lower than in previous reports. Similarly, rates of acute PV reconnection were lower than in controls (11%). AI targets are arbitrary and published targets range from 380 to 400 for the posterior wall and 550 elsewhere. This study used a novel combination of high-power delivered by ST catheters. In this context, an AI target of 400 for the posterior wall and 500 elsewhere led to high rates of first-pass PVI and low rates of acute PV reconnection.

### 4.5. First-Pass Pulmonary Vein Isolation

An earlier study displayed increased efficacy of AI-guided catheter ablation while having comparable safety to non-AI catheter ablation [10]. Chen et al. [38] indicated that AI-guided high-power (50 W) ablation increases first-pass PVI rates. Leshem et al. [13] compared ablation using 90 W for 4 seconds to 25 W for 20 seconds. The 90 W/4-second ablation resulted in full-thickness lesions with no gaps in all cases, whereas the 25 W/20-second ablation resulted in some partial-thickness lesions and many gaps between lesions. At 25 W for 20 seconds, irrigation of the catheter tip seemed to cause “endocardial sparing,” thought to be a failure to create scar because of cooling of the endocardium by irrigation before resistive heating can destroy the tissue. In the present animal study experiment, use of higher power was associated with larger maximum diameter and more thorough tissue necrosis. Greater size and better consistency of the created tissue necrosis may explain why high-power increases procedure efficiency by ensuring more first-pass PVI and fewer reconnections at 20 minutes.

### 4.6. Acute PV Reconnections

Durability of PVI is important to procedural success; both acute and late PV reconnection have been associated with AF recurrence [5, 39]. In a study [14] using an open irrigated-tip catheter, patients undergoing ablation at 50 W vs. 35 W had greater freedom from AF (82% vs. 66%). The idea of the “weakest link” predicting sites of reconnection was described recently by El Haddad and colleagues [40], who found that sites of reconnection were associated with poor lesion depth and lack of contiguous lesion sets. In addition, Dhilon et al. [41] found reduced operative time and reduced acute PV reconnection in patients with paroxysmal atrial fibrillation who underwent AI-guided high-power ablation. As such, the present one documented fewer acute PV reconnections in the high- vs. standard-power group, and in an animal model, higher power caused more thorough tissue necrosis thereby precluding cell restoration and reducing acute pulmonary vein connection.

### 4.7. Complications

HPSD RF delivery is thought to destroy tissue, mostly through local resistive heating, which occurs early during an RF application, by avoiding the distant conductive heating tissue damage that predominates later during long RF applications. In freshly killed porcine ventricles, Goyal et al. [20] showed that the time to create a 4 mm deep lesion was 20 seconds for 20 W ablations and only 6–7 seconds for 50 W ablations, which suggested that high-power, short-duration RF applications might help reduce collateral injury. Bhaskaran et al. [17] showed that 50 W and 60 W ablations for 5 seconds achieved transmural lesions and were safer than 40 W ablations for 30 seconds. The incidence of steam pops was 8% in the 40 W/30-second ablations vs. none in the 50 W and 60 W ablations for 5 seconds. Winkle et al. [18] compared the use of open irrigated-tip catheters at 50 W for short durations of 3-10 seconds at each site to lower power applied for 25-40 seconds at each site. 50 W ablations had longer-term freedom from AF and shorter procedural, fluoroscopy times without an increase in complications. Winkle et al. [42] examined the complication rates of 4 experienced centers performing AF ablations at RF powers from 45-50 W for 2-15 seconds per lesion while power was reduced to 35 W for 20 seconds, AF ablations can be performed at 45–50 W for short durations with very low complication rates. Our clinical results cannot provide definitive information (for example using esophageal temperature monitoring) on whether high-power, short-duration lesions were safer than low-power energy delivered for a longer time. However, our histological results confirmed shallower tissue lesions with high-power than low-power ablation, with shorter ablation time reflecting shorter time for catheter to attach to the atrial wall tissue, thus leading to higher safety. In addition, the extremely low complication rate may be reassuring for using 40 W for short durations in left atrium, even posterior wall and may encourage considering use of short-duration, higher-power RF ablations to take advantage of the reduction in procedural, fluoroscopy, and total RF energy delivery times.

### 4.8. Limitations

Although the results of this study are encouraging, their robustness is limited by several factors. First, degree of esophageal injury during ablation is unclear because all patients were treated under local anesthesia and could not tolerate esophageal temperature monitoring, and no postoperative endoscopic examination was performed. Second, the relatively fixed AI values used may be insufficient or excessive for some patients, especially for thin women. Third, because ST was used instead of Smart Touch Surround Flow (STSF) catheter, there is a small amount of scab at the catheter tip during the 50 W ablation in the animal study, for which, 50 W was not selected for ablation in clinical research. Fourth, after a year, there was a similar sinus rhythm maintenance rate after ablation with 30 W and 40 W which may be because the numbers in each group were probably too small to look at a real difference in these two techniques. Fifth, the animal study is carried out in ventricles while the human study is in atrial. There may be a lack of consistency.

## 5. Conclusions

In the present study of high-power ablation, use of guidance by AI, which provides a rational local endpoint allowing for a tailored short-duration radiofrequency application associated with optimized lesion metrics, translated into shorter procedural time and improved acute efficacy, without compromising safety profile and long-term outcomes relative to standard-power ablation.

## Figures and Tables

**Figure 1:** AI-guided ablation injury. VISITAGs placement with distance measure tool.

**Figure 2:** Ventricular lesions obtained with constant AI of 500 and with 50 W, 40 W, or 30 W of power output. (a) By visual inspection, increasing power was associated with larger lesion maximum diameter (green line) and deeper tissue necrosis (red line), with boundaries of tissue lesion and necrosis becoming clearer. (b–d) Lesions (green line) and necrosis (red line) generated with 30 W, 40 W, and 50 W were examined under 20× amplification; under 400× magnification at 1 mm from the ablation catheter tip in panels B1 (mainly basophilic changes of connective tissue with least myocardial cell changes and nuclear pyknosis), C1 (small number of myocardial cells with fuzzy sarcoplasm, no horizontal stripes and nuclear pyknosis), and D1 (largest number of affected myocardial cells); and under 200× magnification at 3 mm from the ablation catheter tip in panels B2 (no basophilic changes of fibrous connective tissue), C2 (basophilic changes only around cells), and D2 (basophilic changes around the blood vessels and cells).

**Figure 3:** Percentage of total number of RF lesions by average CF ranges.

**Figure 4:** Ablation time per point throughout PV.

**Figure 5:** Energy delivery per point throughout PV.

**Figure 6:** Distribution of contact-force throughout PV.

**Figure 7:** Ablation time throughout PV.

**Table 1:** Sources of drugs and equipment.

Name	Scientific name	Specification	Manufacturer	Approval number	Country
Lidocaine		2 ml/4 mg	Linyi Chenghui Pharmaceutical Co., Ltd.	SFDA approval number H37023396	China
Fentanyl		2 ml:0.1 mg	Jiangsu Nhwa Pharmaceutical Co., Ltd.	SFDA approval number H20113509	China
6F decapolar catheter	Multipolar diagnostic catheter	—	Biosense Webster	—	Diamond Bar, USA
Multipolar mapping catheter	Pentaray, Biosense Webster	—	Biosense Webster	—	Diamond Bar, USA
3.5 mm tip open-irrigated contact force-sensing catheter	ThermoCool Smart Touch (ST)	—	Biosense Webster	—	South Diamond Bar, USA

**Table 2:** Swine ventricular lesion and necrosis characteristics.

Variable	50 w	40 w	30 w
Ablation time per point, s∗	20.00 ± 1.10	27.78 ± 9.72	44.83 ± 9.83
Ventricular lesion impedance drop, *Ω*∗	13.5 ± 1.87	9.11 ± 1.54	6.17 ± 0.98
Energy delivery per point, J∗	992.30 ± 54.33	1085.10 ± 45.02	1337.0 ± 24.42
Ventricular tissue lesion depth, mm∗	3.95 ± 0.16	4.38 ± 0.13	5.06 ± 0.16
Ventricular tissue necrosis depth, mm∗	3.15 ± 0.18	2.71 ± 0.17	2.42 ± 0.13
Ventricular tissue lesion width, mm∗	9.08 ± 0.15	8.42 ± 0.18	7.81 ± 0.15
Ventricular tissue necrosis width, mm∗	5.58 ± 0.18	5.18 ± 0.16	3.94 ± 0.17

∗All *p* values < 0.001.

**Table 3:** Clinical characteristics.

Variable	Study group High-power (*n* = 50)	Control group Standard power (*n* = 50)	*p* value
Age, y∗	64.4 ± 9.45	64.9 ± 8.62	0.862
Male	34 (68)	32 (64)	0.673
LV ejection fraction, %	64.74 ± 4.46	61.9 ± 5.40	0.08
Left atrial size, mm	40.65 ± 5.87	42.85 ± 3.10	0.147
Hypertension	22 (44)	26 (52)	0.423
Diabetes mellitus	6 (12)	8 (16)	0.564
Body mass index	21.27 ± 1.88	21.04 ± 2.65	0.749
Prior stroke/transient ischemic attack	8 (16)	10 (20)	0.603
Coronary artery disease *n*	14 (28)	12 (24)	0.648
CHADS2 score	2.1 ± 0.64	1.95 ± 0.80	0.504
CHA2DS2-VASC score	3.4 ± 1.14	3.15 ± 1.04	0.474
Obstructive sleep apnea	6 (12)	7 (14)	0.766
Dilated cardiomyopathy	3 (6)	3 (6)	1

Data are presented as mean ± SD or *n* (%).

**Table 4:** Procedural characteristics.

Variable	Study group High power (40 W) *n* = 50	Control group Standard power (30 W); *n* = 50	*p* value
Procedure time, min	56.54 ± 1.81	76.55 ± 2.34	<0.001
Right encirclement procedure time, min	30.92 ± 1.31	38.33 ± 3.06	<0.001
Left encirclement procedure time, min	25.83 ± 1.12	37.92 ± 1.24	<0.001
Right encirclement points, *n*	51.25 ± 2.45	49.08 ± 3.58	0.1
Left encirclement points, *n*	44.42 ± 1.44	45.00 ± 1.91	0.407
Total ablation time, min	35.85 ± 14.87	51.01 ± 17.99	<0.001
Contact-force, g∗	12.07 ± 5.34	11.85 ± 5.40	0.523
Ablation time per point, s	22.64 ± 9.39	32.56 ± 11.48	<0.001
Energy delivery per point, J∗	909.02 ± 354.57	1045 ± 376.60	<0.001
Impedance drop per point, *Ω*∗	10.13 ± 1.624	6.57 ± 1.012	<0.001
First-pass PVI	87 (87)	72 (72)	<0.01
Reconnection after 20 min	22 (11)	46 (23)	<0.01
Groin hematoma	1	1	1
Tamponade	0	0	1
Periprocedural stroke	0	0	1
Esophageal fistula	0	0	1
Sinus rhythm at 12 months	46 (92)	42 (84)	0.22

Data are presented as mean ± SD or *n* (%).

## Data Availability

The datasets generated during and/orc analyzed during the current study are not publicly available, but are available from the corresponding author on reasonable request.

## Additional Points

*Posted History*. A preprint has previously been published [43]. The link is as follows https://www.researchsquare.com/article/rs-21367/v2.
